The article "Analysis of Diversified Radio and Television Data Based on Adaptive Least Squares Support Vector Machine" was published in 2022. Journal: Comput Intell Neurosci.

# Analysis of Diversified Radio and Television Data Based on Adaptive Least Squares Support Vector Machine

**DOI:** 10.1155/2022/4235088

**Published:** 2022-07-05

**Authors:** Jing Liu, Minnan Cang

**Affiliations:** ^1^College of Liberal Arts, Chifeng University, Neimenggu 024000, China; ^2^Xi'an University of Technology the School of Art and Design, Xi'an 710000, China

## Abstract

Under the current big data background, the training mode of radio and television director technology is obsolete, and the technical means do not meet the needs of modern development. In this article, a self-adaptive multivariate data statistical model of radio and television directors based on the least squares support vector machine is proposed, which combines the students' views with the diversified teaching methods and teaching contents needed by university teachers in the process of vocational education and television education. This article applies the technology integration degree measurement, market integration degree measurement, business integration degree measurement, and integration degree comprehensive analysis to analyze the data of major video websites and major radio and television media. It is found that the market share of major radio and television media is increasing, and the number of broadcasts of major video online stores is also excellent.

## 1. Introduction

According to China's demand for talents in radio and television industry and the status of education professionals, the director of experimental teaching of radio and television specialty should actively introduce the advanced teaching concept of postmodernism; evaluate and innovate from the aspects of experimental teaching mode, process, method, and behavior; build an experimental teaching system with the characteristics of postmodern teaching theory; and cultivate the innovative spirit and practical ability of radio and television art complex [1]. With the continuous development of new media technology, the market demand for employment is gradually increasing, but the market competition is becoming increasingly fierce. The development of radio and television specialty in China needs more radio and television professionals, and the requirements for talents' skills and quality are also improved. With the rapid development of new media, the demand for applied talents of radio and television director specialty is gradually increasing [2]. A new discrete particle swarm optimization method is proposed to induce rules from discrete data. The proposed algorithm initializes the population by considering the discrete nature of the data. It assigns different fixed probabilities to the current, local, and global optimal positions. Based on these probabilities, each member of the population iteratively updates its position [3]. The explicit model-based approach to phylogenetic analysis of discrete morphological data opens up several new research approaches, including combined data likelihood analysis (morphological + sequential data), likelihood ratio test, and Bayesian analysis [4]. Linear hybrid models have become the main parameterization tool for analyzing continuous longitudinal data. This article shows how to implement different methods in the SAS software package [5]. Data interpolation is created under two models: multivariate normal model with rounding and discrete model with conditional designation. JM method introduces deviation in reference curve, while FCS does not. This article concludes that FCS is a useful and easy-to-apply flexible alternative to JM [6] when convenient and realistic joint distribution cannot be specified. Chameleon algorithm technology focuses on finding clusters in datasets and detailed information of its main functions, dynamic modeling information of chameleon and comparison between interconnectivity and similarity (limitations of traditional clustering algorithms) [7]. This article evaluates the changing role of dynamic modeling in understanding and discrete dynamic modeling of diversified adaptive data for broadcast and television directors. It discusses new modeling tools for problem scoping and consensus building among a wide range of stakeholders and describes four case studies where dynamic modeling has been used to collect and organize data, synthesize knowledge, and build consensus on the management of complex systems [8]. Two methods to solve the problem of dynamic allocation and route guidance are studied: first, the optimal control method to realize the optimization of a dynamic system or user; second, to establish the feedback concept of dynamic user optimal conditions [9]. Landscape and physical environment shape migration schedules and affect people's ability to interpret patterns observed during stopovers. Modeling these factors may lead to new insights into migration adaptation in heterogeneous environments [10]. Scale dependence and spatiotemporal dynamics are the two issues that underpin the considerable attention that modelers and statisticians now devote to the quantitative study of ecological edges and boundaries. We introduced the links between methods for demarcating boundaries, monitoring boundary changes, and modeling edge-related dynamics. In this process, we clarify the statistical and mathematical methods of ecological edge and boundary research and discuss the important remaining problems in the field of quantitative edge research [11]. In order to adapt to the gradual diversified development, a diversified training mode for graduate students has been formed. At the same time, in order to meet the needs of people's learning and creation in modern society, graduate education presents an international, diversified, modern, and personalized development trend [12]. Their most influential discrete imaging (DT) uses nanoscale technology to generate a large amount of data. Data footprint production (DFR) is a process that uses almost all of given ETF data at a shorter storage speed. His very advanced lossless compressor or classical probability model is very suitable for final application requirements, such as “arbitrary depth” (ABD) solutions and “dynamic data scale, exploring data-related information” [13]. The moving window detection process of discrete data is studied. The probability of detection waiting time and the limit of expected value are derived. The boundary is evaluated for independent and identically distributed zero-Bernoulli test, binomial and Poisson random variables, and two-state stationary Markov chain. The results are applicable to radar detection theory, time-sharing system, and quality control [14]. For goals and training programs, by constructing a scientific curriculum system, establishing characteristic curriculum relations, expanding diversified teaching forms, strengthening innovative practical teaching concepts, and developing digital laboratories and other measures, we can train talents, explore Sino-foreign cooperative training methods suitable for the development of China's digital media design industry, and improve the quality and level of digital media design talents training [15]. The development of big data technology has brought new opportunities and challenges to the development of various industries. The radio and television director industry has been widely favored by the broad masses of the people, and its development is directly related to everyone's daily life. People's daily life can no longer be separated from big data technology, whether it is the TV we watch every day or a mobile phone. They all use the technical support of big data, better demonstrate the skills developed in the data age, and show stronger conditions for the progress and formation of the data age. Therefore, in the current development of education, we must master the technical support of big data, expand the content and form of TV director better, help the content of TV education show more power, and lay a solid foundation for improving the quality of TV director content. In order to better cope with the impact and challenges of the big data era and the relevant requirements for talents in the era of big data, colleges and universities need to implement diversified training modes, cultivate high-skilled and high-quality talents, and provide college students with due guarantee in the ability to use big data technology and the ability to use and build big data technology. It can show the creativity of talents in TV choreography and the significance of TV choreography more deeply, and optimize, improve, and systematically train the existing talent training system, so as to provide talent support for the development of radio and TV choreography industry. Based on this, this article introduces the diversified literacy requirements of radio and television directors in the era of big data and summarizes the diversified training strategies of radio and television directors in the era of big data, so as to better promote the development and technical requirements of TV directors in the era of big data and promote the further formation of talents.

## 2. The Strategy of Cultivating Diversified Applied Talents of Radio and Television Directors

### 2.1. Cultivating Students' Ability to Analyze and Control Big Data

In the era of big data, the most important thing is information. The available material found in several lines of information is ability. According to big data, it is skill to analyze the development trend of events. Using big data to guide public opinion to develop in the expected direction depends on skills.

If you want to create excellent radio and television programs, you can select useful information on the big data platform and then recombine the useful information. At present, the idea of many reality shows is to find out what the audience likes to watch through big data analysis and then summarize and extract useful information for innovative creation, which is the source of the embryonic form of reality shows.

It is necessary to cultivate students' ability of information prediction and early warning. In the era of big data, a large amount of information is released all the time. As a radio and television-related worker, he must have the form of predicting the future development through this information. When some events are constantly fermenting, he should be aware of the seriousness of the situation in time, so as to make preventive plans in advance.

Finally, it is the ability to use big data to guide the trend of public opinion. Choreographers need to put forward their views in a timely manner, which should be novel and attract the attention of a broad audience, so as to make public opinion tilt towards the favorable side.

### 2.2. Curriculum Setting of Diversified Choreography Specialty

The purpose of the curriculum is to increase the content of education. In addition to the original editorial guidance courses, students must broaden their horizons, edit art and news programs, and add data and information courses. Teachers should not only let students stay in the studio and broadcast live, but also go out, use big data to keep abreast of the latest developments, capture creative inspiration, and apply the latest technology and film and television processing technology to their programs. In order to help students learn how to analyze, acquire, edit, and transmit information to capture creative themes, data information courses can be added to break through the bottleneck of choreography and creation and become diversified talents.

### 2.3. Focusing on Cultivating Students' All-Media Thinking Mode

With the popularization of the Internet and the development of information technology, the types and functions of broadcasting are constantly updated, and the program content is gradually diversified. The TV also adds images and text based on video data. In this context, the director talent training strategy should be further refined, focusing on cultivating students' all-media thinking, so that students can choose the most suitable media mode according to the content of radio and television programs and the characteristics of media audiences. At present, different forms of media are developing together. If radio and television students do not have all the media and energy to study professional knowledge, while ignoring literature, society, and nature, they are likely to limit your major and your own development.

### 2.4. Perfecting the Practical Teaching Function of Choreography Specialty

First of all, we can join practical activities in the teaching process of choreography. Practice is the basic work of radio and television director, and it is the materials close to life that are more likely to resonate with the audience, so as to ensure attention and click-through rate. Second, schools can work with major media to provide students with more practical opportunities. After graduation, media work is no stranger to students, which effectively shortens the adjustment time. Schools and media organizations will benefit from this process. Students can help the media analyze and organize information. Schools can take the advantage of big data analysis and visual advantages to gain more practical communication opportunities between schools. The media are more closely linked. In the past teaching activities, students majoring in choreography cannot finish news writing or program creation because they do not have practical materials. With the advent of the era of big data, students have realized their dream of seeing what is going on in the world without leaving home. Students can grasp the current audience's interest trend by analyzing research reports and news information and then summarizing these contents. After analysis and screening, they can provide themselves with complete director materials.

### 2.5. Cultivating Students' Ability to Interpret Radio and Television Programs

Schools can improve students' ability to interact with big data. When cultivating choreographers' storytelling ability, they can use big data to analyze social current affairs, explore the information value behind big data, and use topics that can attract social attention to create big data and create inspiration for their own creative inspiration. At present, topics with high attention in society often come from people's daily life. Topic content with life as the theme and high statistical attention is likely to become radio and television content with less investment and high popularity. The cultivation of this ability is especially suitable for the current choreography major, and stories supported by big data analysis will be more convincing.

## 3. Improvement in Online Adaptive Least Squares Support Vector Machine Algorithm

### 3.1. Online Adaptive Least Squares Support-Oriented Computer Algorithm

Let the sample set be *T*={(*x*_1_, *y*_1_),…, (*x*_*l*_, *y*_*l*_)}, where *x*_*i*_ ∈ *R*^*n*^, *y*_*i*_ ∈ *R*, *i*=1,2,…, *l* constructs the decision function *f*(*x*)=*w*^*T*^Φ(*x*_*i*_)+*b* and use the sample data to solve the objective function of minimizing structural risk, which is expressed as

(1) $$\begin{array}{c} \underset{w,b}{\min}\frac{1}{2}{\left\|w\right\|}^{2}+c\sum_{i=1}^{l}\zeta_{i}^{2}, \end{array}$$

(2) $$\begin{array}{c} y_{i}=w\cdot \Phi \left(x\right)+b+\xi_{i},\;i=1,2,\ldots ,l, \end{array}$$

where Φ(*x*_*i*_) is *x*_*i*_ nonlinear mapping, *w* and *b* are function parameters, *c* is a parameter, and *ξ*_*i*_ is a prediction error.

The above problem can be transformed into formula (3) by using the related Lagrange function:

(3) $$\begin{array}{c} L\left(w,b,\xi ,a\right)=\frac{1}{2}{\left\|w\right\|}^{2}+c\sum_{i=1}^{l}\xi_{i}^{2}-\sum_{i=1}^{l}a_{i}\left(w\cdot \Phi \left(x\right)+b+\xi_{i}-y_{i}\right), \end{array}$$

where *a*=[*a*_1_, *a*_2_,…, *a*_*l*_] is the Lagrange multiplier; *ξ*=[*ξ*_1_, *ξ*_2_,…, *ξ*_*l*_] is the training set prediction error vector. According to the optimization conditions, formula (4) can be obtained as

(4) $$\begin{array}{c} \frac{\partial L}{\partial w}=0,\frac{\partial L}{\partial b}=0,\frac{\partial L}{\partial \xi_{i}}=0,\frac{\partial L}{\partial a_{i}}=0. \end{array}$$

Formula (5) can be solved as

(5) $$\begin{array}{c} \left\{\begin{array}{c} w=\sum_{i=1}^{l}a_{i}\Phi \left(x_{i}\right),\\ \sum_{i=1}^{l}a_{i}=0,\\ 2c\xi_{i}=a_{i}. \end{array}\right. \end{array}$$

Formula (6) can be obtained by substituting formula (5) into formula (2).

(6) $$\begin{array}{c} y_{i}=\sum_{j=1}^{l}\left(a_{j}\cdot \langle \Phi \left(x_{i}\right),\Phi \left(x_{j}\right)\rangle \right)+b+\frac{1}{2c}a_{i}. \end{array}$$

If *K*(*x*_*i*_, *x*_*j*_)=〈Φ(*x*_*i*_), Φ(*x*_*j*_)〉 is defined as a kernel function, formula (6) is transformed into a set of linear equations, which is expressed as

(7) $$\begin{array}{c} \left[\begin{array}{ccccc} 0 & 1 & 1 & \cdots & 1\\ 1 & K\left(x_{1},x_{1}\right)+\frac{1}{2c} & K\left(x_{1},x_{2}\right) & \cdots & K\left(x_{1},x_{l}\right)\\ 1 & K\left(x_{2},x_{1}\right) & K\left(x_{2},x_{2}\right)+\frac{1}{2c} & \cdots & K\left(x_{2},x_{l}\right)\\ \vdots & \vdots & \vdots & \ddots & \vdots \\ 1 & K\left(x_{l},x_{l}\right) & K\left(x_{l},x_{2}\right) & \cdots & K\left(x_{l},x_{l}\right)+\frac{1}{2c} \end{array}\right]\cdot \left[\begin{array}{c} b\\ a_{1}\\ a_{2}\\ \vdots \\ a_{l} \end{array}\right]=\left[\begin{array}{c} 0\\ y_{1}\\ y_{2}\\ \vdots \\ y_{l} \end{array}\right]. \end{array}$$

To cause

(8) $$\begin{array}{c} H=\left[\begin{array}{cccc} K\left(x_{1},x_{1}\right)+\frac{1}{2c} & K\left(x_{1},x_{2}\right) & \cdots & K\left(x_{1},x_{l}\right)\\ K\left(x_{2},x_{1}\right) & K\left(x_{2},x_{2}\right)+\frac{1}{2c} & \cdots & K\left(x_{2},x_{l}\right)\\ \vdots & \vdots & \ddots & \vdots \\ K\left(x_{l},x_{1}\right) & K\left(x_{l},x_{2}\right) & \cdots & K\left(x_{l},x_{l}\right)+\frac{1}{2c} \end{array}\right],\\ y={\left[y_{1},y_{2},\ldots ,y_{l}\right]}^{T}, \end{array}$$

where *e*=[1, ⋯,1]_1×*l*_^*T*^; *a*=[*a*_1_, *a*_2_, ⋯,*a*_*l*_]^*T*^.

Formula (8) can be derived as

(9) $$\begin{array}{c} \left\{\begin{array}{c} a=H^{-1}y-H^{-1}e\cdot \frac{e^{T}H^{-1}y}{e^{T}H^{-1}e},\\ b=\frac{e^{T}H^{-1}y}{e^{T}H^{-1}e}. \end{array}\right. \end{array}$$

To solve the decision function, formula (8) is substituted into formula (9), which isexpressed as

(10) $$\begin{array}{c} f\left(x\right)=\sum_{j=1}^{l}a_{j}K\left(x,x_{j}\right)+b. \end{array}$$

When the prediction of the model has a large deviation, it is updated online.

First, the sample point *i* closest to the current new sample {*x*_*new*_, *y*_*new*_} is found in the original sample space, as in formula (10).

(11) $$\begin{array}{c} i=\arg\left(\underset{k=1,\cdots l}{\min}\left\|x_{\text{new}}-x_{k}\right\|\right). \end{array}$$

Second, the row and column corresponding to the *i* sample in Matrix *H* are exchanged with the last row and column to obtain *H*_1_, as shown in formula (11).

(12) $$\begin{array}{c} H_{1}=I_{Ri↔Rl}HI_{Li↔Ll}, \end{array}$$

where $H_{1}=\left[\begin{array}{ccccc} K\left(x_{1},x_{1}\right)+1/2c & \cdots & K\left(x_{1},x_{l}\right) & \cdots & K\left(x_{1},x_{i}\right)\\ \vdots & \ddots & \vdots & \ddots & \vdots \\ K\left(x_{l},x_{1}\right) & \cdots & K\left(x_{l},x_{l}\right)+1/2c & \cdots & K\left(x_{l},x_{i}\right)\\ \vdots & \ddots & \vdots & \ddots & \vdots \\ K\left(x_{l},x_{1}\right) & \cdots & K\left(x_{i},x_{l}\right) & \cdots & K\left(x_{i},x_{i}\right)+1/2c \end{array}\right]$; *I*_*Ri*↔*Rl*_ and *I*_*Li*↔*Ll*_ represent row *i* and *l* interchange and column *i* and *l* interchange of identity matrix, respectively. *I*_*Ri*↔*Rl*_=*I*_*Li*↔*Ll*_=*I*_*Ri*↔*Rl*_^−1^=*I*_*Li*↔*Ll*_^−1^.

To cause

(13) $$\begin{array}{c} H_{1}=\left[\begin{array}{cc} G & g_{1}\\ g_{1}^{T} & k_{1} \end{array}\right],\\ k_{i}=K\left(x_{i},x_{i}\right)+\frac{1}{2c},\\ g_{i}={\left[K\left(x_{1},x_{i}\right),\ldots ,K\left(x_{i-1},x_{i}\right),K\left(x_{l},x_{i}\right),K\left(x_{i+1},x_{i}\right),\ldots ,K\left(x_{l-1},x_{i}\right)\right]}_{l\times 1}^{T}. \end{array}$$

Because $A^{-1}={\left[\begin{array}{cc} A_{11} & A_{12}\\ A_{21} & A_{22} \end{array}\right]}^{-1}=\left[\begin{array}{cc} A_{11}^{-1}+A_{11}^{-1}A_{12}B^{-1}A_{21}A_{11}^{-1} & -A_{11}^{-1}A_{12}B^{-1}\\ -B^{-1}A_{21}A_{11}^{-1} & B^{-1} \end{array}\right]$, of which *B*^−1^=*A*_22_ − *A*_21_*A*_11_^−1^*A*_12_, so

(14) $$\begin{array}{c} H_{1}^{-1}={\left[\begin{array}{cc} G & g_{i}\\ g_{1}^{T} & k_{i} \end{array}\right]}^{-1}=\left[\begin{array}{cc} G^{-1}+G^{-1}g_{i}r_{i}^{-1}g_{1}^{T}G^{-1} & -G^{-1}g_{i}r_{i}^{-1}\\ -r_{i}^{-1}g_{i}^{T}G^{-1} & r_{i}^{-1} \end{array}\right]=\left[\begin{array}{cc} G^{-1} & 0\\ 0 & 0 \end{array}\right]+\left[\begin{array}{cc} G^{-1}g_{i}r_{i}^{-1}g_{1}^{T}G^{-1} & -G^{-1}g_{i}r_{i}^{-1}\\ -r_{i}^{-1}g_{1}^{T}G^{-1} & r_{i}^{-1} \end{array}\right], \end{array}$$

where *r*_*i*_=*k*_*i*_*g*_*i*_^*T*^*G*^−1^*g*_*i*_.

At the same time, we might as well make:

(15) $$\begin{array}{c} H_{1}^{-1}=\left[\begin{array}{cc} G^{-1} & 0\\ 0 & 0 \end{array}\right]+\left[\begin{array}{cc} {\tilde{h}}_{11} & {\tilde{h}}_{12}\\ {\tilde{h}}_{21} & {\tilde{h}}_{22} \end{array}\right]=\left[\begin{array}{cc} h_{11} & h_{12}\\ h_{21} & h_{22} \end{array}\right], \end{array}$$

where ${\tilde{h}}_{11}=G^{-1}g_{i}r_{i}^{T}G^{-1};{\tilde{h}}_{12}=-G^{-1}g_{i}r_{i}^{T};{\tilde{h}}_{21}=-r_{i}^{-1}g_{i}^{T}G^{-1};{\tilde{h}}_{22}=r_{i}^{-1};G^{-1}=h_{11}-{\tilde{h}}_{11}=h_{11}-h_{12}h_{22}^{-1}h_{21}$.

Therefore, *G*^−1^ can avoid direct inversion of matrix.

The parameters related to the new sample are calculated to replace the original wrong data.

(16) $$\begin{array}{c} g_{\text{new}}={\left[K\left(x_{1},x_{\text{new}}\right),\ldots ,K\left(x_{I-1},x_{\text{new}}\right),K\left(x_{l},x_{\text{new}}\right),K\left(x_{i+1},x_{\text{new}}\right),\ldots ,K\left(x_{l-1},x_{\text{new}}\right)\right]}_{l\times 1}^{T},\\ k_{\text{new}}=K\left(x_{\text{new}},x_{\text{new}}\right)+\frac{1}{2c},\\ r_{\text{new}}=k_{\text{new}}-g_{\text{new}}^{T}G^{-1}g_{\text{new}}\text{,}\\ So:H_{2}^{-1}=\left[\begin{array}{cc} G^{-1}+G^{-1}g_{\text{new}}r_{\text{new}}^{-1}G^{-1} & -G^{-1}g_{\text{new}}r_{\text{new}}^{-1}\\ -r_{\text{new}}^{-1}g_{\text{new}}^{T}G^{-1} & r_{\text{new}}^{-1} \end{array}\right]. \end{array}$$

Finally, the updated decision function coefficient can be obtained from the following equation:

(17) $$\begin{array}{c} \left\{\begin{array}{c} \hat{a}=H_{2}^{-1}\hat{y}-H_{2}^{-1}e\cdot \frac{e^{T}H_{2}^{-1}\hat{y}}{e^{T}H_{2}^{-1}e},\\ \hat{b}=\frac{e^{T}H_{2}^{-1}\hat{y}}{e^{T}H_{2}^{-1}e}, \end{array}\right. \end{array}$$

where $\hat{y}={\left[y_{1},\ldots ,y_{i-1},y_{l},y_{i+1},y_{new}\right]}^{T}$.

## 4. Fusion Degree Measurement

### 4.1. Measurement of Technology Integration Degree

1. This article collates the investment scale of the central nervous system and broadband fees from 2012 to 2016 of four major video websites and four major radio and television media (Table 1)
2. In order to better reflect the classification of advertising revenue, the classification data of major video websites and major radio and television media are sorted out (Table 2)
3. Sample unit HI value calculation (Table 3)
4. Evaluation of fusion degree

From Table 4, the HI values of CND and broadband fee investment scale of major video websites and major radio and television media from 2012 to 2016 are substituted into different integration degree interval values. It can be seen that the technology integration degree of major video websites and major radio and television media is generally low, among which, in 2012, 2013, 2015, and 2016, it was in a low-to-medium integration state, and in 2014, it was relatively good and in a moderate integration state.

According to the HI value of CND and broadband fee investment scale of major video websites and major radio and television media in each year, the change chart of CND and broadband fee investment HI value from 2012 to 2016 is drawn, as shown in Figure 1.

### 4.2. Measurement of Market Integration Degree

#### 4.2.1. Collation of Sample Unit Data

According to the statistics of State Administration of Press, Publication, Radio, Film and Television in 2016, this article collates the radio and television advertising revenue of four major video websites, including Unity group, Tencent video, Sohu video, and Iqiyi, and four major radio and television media, including CCTV, China National Radio, China Radio International, and Hunan Radio and Television Station, from 2012 to 2016 (Table 5).

In order to better reflect the classification of advertising revenue in major video websites and major radio and television media, the classified data of four major video websites, such as Unity group, Tencent video, Sohu video, and Iqiyi, and four major radio and television media, such as CCTV, China National Radio, China Radio International, and Hunan Radio and Television Station, are sorted out (Table 6).

#### 4.2.2. Sample Unit HI Value Calculation

HI value of advertising revenue is given in Table 7.

#### 4.2.3. Evaluation of Fusion Degree

According to the HI value of advertising revenue calculated in Table 7, the HI value of advertising revenue of major video websites and major radio and television media from 2012 to 2016 is substituted into different integration degree interval values, respectively, and it can be seen that the market integration degree of major video websites and major radio and television media is in a low integration state (Table 8).

According to the HI value of advertising revenue of major video websites and major radio and television media in each year, the change chart of advertising revenue HI value from 2012 to 2016 is drawn, as shown in Figure 2.

### 4.3. Measurement of Service Convergence Degree

Collation of sample unit data. From 2012 to 2016, the PC page playback, PC client playback, mobile page playback, and mobile client playback are given in Tables 9–12, respectively.

According to Tables 9–12, we calculate the average number of times that Heyi group, Tencent video, Sohu video, and Iqiyi play on PC page side, PC client side, mobile page side, and mobile client side, and then draw a histogram as shown in Figure 3.

In order to better observe and judge the abovementioned major video websites and major radio and television media from 2012 to 2016, the overall classification of playing platforms such as PC page side, PC client side, mobile page side, and mobile client side, the overall development trend and development stage of major video websites and major radio and television media in terms of business integration degree are calculated. Figure 3 shows the video development of four different platforms in different years. Mobile clients have developed rapidly, and in 2016, mobile clients are almost the sum of other platforms. On the whole, the development of PC as a media is slow, and the basic processing stops. According to the relevant data calculated in Tables 9–12 above, this article analyzes and summarizes the classified data of major video websites and major radio and television media (Tables 13–16).

According to Tables 13–16, we calculate the average number of times played by major video websites and major radio and television media on PC page side, PC client side, mobile page side, and mobile client side, and then draw a histogram as shown in Figure 4.

Sample unit HI value calculation: according to the calculation model of Herfindahl index method, the HI values of PC page playback, PC client playback, mobile page playback, and mobile client playback of major video websites and major radio and television media from 2012 to 2016 are calculated, as given in Tables 17–20.

According to Tables 17–20, we calculate the average HI values of the playing times of major video websites and major radio and television media on PC page side, PC client side, mobile page side, and mobile client side, and then draw a histogram as shown in Figure 5.

Evaluation of fusion degree: according to Tables 17–20, the playback frequency of major video websites and major radio and television media on PC page side, PC client side, mobile page side, and mobile client side was in a low convergence range from 2012 to 2016, and only in 2016, the playback frequency on PC page side showed moderate convergence, among which major video websites were superior to major radio and television media as a whole.

The smaller the HI value, the higher the degree of industrial integration, and the greater the HI value, the lower the degree of integration. Through comparative analysis in Table 21, the overall integration of radio and television media and new media is low. Among them, the performance of technology integration, market integration, and business integration of radio and television media lags far behind the new media industry. The new media based on the Internet undoubtedly has great communication power, influence, and mobilization power and has been in a comprehensive leading state in technology, market, and business, occupying the strategic highland of various media. Compared with the telecommunications industry, the radio and television media as a whole are dwarfed.

Generally speaking, the media integration of radio and television industry is divided into three levels. First, the initial integration, that is, the programs are uploaded to the network platform and transformed into terminals suitable for mobile phones, desktops, and tablet computers by means of disassembly, packaging, and reorganization, so as to adapt to network communication. The second is moderate integration, that is, in news collection and editing, news materials are collected through handheld terminals, desktops, and radio and television channels, and news events are broadcasted by editors on new media platforms and then made into audio and video programs for broadcasting on radio and television stations. This way can realize the linkage transmission mechanism of the same news content in different carriers such as radio and television, WeChat Weibo, network, car and outdoor TV, newspapers, and periodicals. Third, deep integration, through cooperation with professional video websites and portal websites, expands the transmission path of radio and television through advantageous network platforms, so as to increase the penetration rate and influence of radio and television programs. At present, although the vast majority of radio and television stations above the prefecture level have set up video and audio websites, and some have set up Weibo accounts, WeChat official account, and developed boutique program applications and clients, they are still in the initial and moderate integration stage as a whole. As the market continues to mature and become more perfect, social capital will become more important and the competition between industries will intensify further, especially with the diversification of TV audience program signal receiving methods. With the increase in traditional media and the emerging audio and media integration services, users' consumption habits change gradually, and cable TV users turn to IPTV, OTT, video websites, and other new media. The market share of cable TV is declining day by day, and the competitive pressure of radio and television industry will be increasing.

#### 4.3.1. Degree of Technology Integration

On the one hand, we can see that the degree of technology integration is better than the degree of market integration and business integration as a whole, and the overall performance is getting better from 2012 to 2016, which reflects the efforts made by radio and television media in technology integration to a certain extent. For example, CCTV is committed to China's video cloud service platform; integrates CCTV news, mobile TV platform, and CCTV audio-visual and other new media platforms; promotes the preinstallation of CCTV audio-visual and news clients and China Mobile cooperative models; establishes collaborative linkage between different receiving terminal platforms; and distributes content to desktop computers, tablet computers, mobile phones, televisions, outdoor large screens, and other terminals. China National Radio connects the car network and the mobile Internet market by building a China broadcasting cloud platform. From the analysis of the proportion of major video websites and major radio and television media (CND and broadband fee investment in advertising revenue in Table 22), it can be seen that major radio and television media still attach great importance to the investment in technology, and the related investment in 2014 and 2016 even exceeded the total advertising revenue of that year. From 2012 to 2016, CCTV, China National Radio, China Radio International, and Hunan Radio and Television have invested a total of 2.899 billion yuan in CND and broadband. The four major video websites have invested a total of 14.4 billion yuan in CND and broadband, with a difference of 4.97 times. Among them, the investment of any of the four major video websites in CND and broadband far exceeds the total investment of the four major radio and television media. The capital strength of new media and the high investment in technology integration can be seen. Generally speaking, some radio and television organizations have not paid enough attention to the subversive impact brought by media convergence, and still muddle along in the hotbed of vested interests of radio and television; and some simply transplant traditional radio and television programs to websites and new media platforms, but do not interpret the programs as the suitable broadcasting form and customer acceptance habit paradigm for the Internet, especially the mobile Internet.

#### 4.3.2. Degree of Market Integration

Advertising revenue is a barometer of the media market. In the new media market, four major video websites have occupied a dominant position, among which the advertising revenue in 2016 was 15.5 billion yuan, accounting for 41% of the national related advertising revenue of 37.5 billion yuan. On the other hand, the related advertising revenue of the four major radio and television media in 2016 was 1.25 billion yuan, accounting for only 3.33% of the national related advertising revenue. It is precisely because of the versatility of assets brought about by technological progress and media convergence that once news and other audio and video programs are produced, due to the noncompetitive sharing and weak increase in reproduction costs, the production cost is saved, and due to the pressure of external competition, the price competition is obvious. Compared with the business packages of telecommunication departments that provide three-in-one services of TV, telephone, and Internet, the price competitive disadvantage of radio and television media is self-evident and directly affects the share of advertising revenue. Generally speaking, affected by administrative monopoly factors, the market behavior of radio and television industry is extensive, and the efficiency of market resource allocation needs to be further improved. It is necessary to make rational use of radio and television resources, further reduce market access, and effectively form a good competitive situation. With the in-depth integration with new media, the editing process and organizational structure of radio and television media will undergo profound changes; form a production process of collecting multimedia generation and multichannel and multiplatform information release; realize collaborative communication and integrated production; improve the productivity of various departments; promote the improvement in the economic benefits of the whole media; realize the multiple appreciation of media assets and resources; realize the full utilization and reallocation of common elements and common assets; change the weak cost increase between radio and television media into the weak cost increase within the new media; and realize the improvement in market performance. Of course, radio and television media have also made a lot of efforts in market integration and actively explore new ways of marketing on the basis of continuing to adhere to the principle of “content is king.”

#### 4.3.3. Degree of Business Integration

The performance of the three integration indicators is the worst, and there is a slow upward trend in the later period, indicating that the business integration of the two industries is gradually deepening, but the pace is relatively slow. Of course, the contribution of major video websites in this respect is major. As given in Table 23, the total playing frequency of major video websites on PC page side, PC client side, mobile page side, and mobile client side has increased rapidly, reaching 1,673.101 billion times in 2016, which is 11.6 s times of the 144.252 billion times of major radio and television media. Although the total broadcast frequency of major radio and television media is also increasing greatly, it is generally inadequate, especially the broadcast frequency of PC clients, which is basically blank in China National Radio, China Radio International, and Hunan TV Station. Media convergence will give birth to a large number of new products and services, which not only enrich the audience's choices, but also become the tools and fields for radio and television media to compete with new media. Audience's choice of radio and television programs is voted by remote control. When the program is broadcast, netizens can express their views to the contestants, and the TV screen can also present the opinions of Weibo netizens in real time, so as to realize the three-screen interaction among TV screen, mobile phone screen, and computer screen, which meets the audience's opinion expression and interaction needs and successfully attracts young network users to the TV screen. Hunan Satellite TV pays attention to the integration with its own new media to produce programs and realizes the deep integration of traditional media and new media content production by means of joint research and planning, separate organization and implementation, unified arrangement and production, and external integration and presentation.

The data in above tables are missing, mainly because there is no corresponding data source. Some media have not been applied on the Internet before, and many data cannot be verified or have no relevant data application.

## 5. Conclusion

Big data endows the radio and television director industry with new characteristics. In order to meet the needs of the times and find the space for students to survive and develop in surgical guidance, colleges and universities need to transform their skills, adopt diversified open teaching methods, optimize the existing professional personnel training mode, rationally organize radio and television teacher courses, and form a double-qualified team. Strong teachers cultivate data, better cultivate more radio and television directors to meet the development needs of the big data era, contribute to the sustainable and long-term development of cultural enterprises, and study and formulate a brand-new talent training strategy. The next step is to analyze the application characteristics of different media in communication effect and commercial value. From different business recommendations, the media application in precision business model has a new application prospect, which is suitable for the method proposed in this article and needs further verification.

## Figures and Tables

**Figure 1:** HI value change chart.

**Figure 2:** Change chart of HI value of advertising revenue.

**Figure 3:** Comparison of average playback times from 2012 to 2016.

**Figure 4:** Comparison of average playback times from 2012 to 2016.

**Figure 5:** Comparison of average HI value of play times from 2012 to 2016.

**Table 1:** Investment scale of CND and broadband fees of major video websites and major radio and television media.

Unit	CND and broadband fee investment scale (10,000 yuan)				
	2012	2013	2014	2015	2016
Unity group	44,586.84	52,708.30	74,000.15	80,923.80	160,833.00
Tencent video	15,432.12	32,431.00	80,000.00	100,000.00	213,960.00
Sohu video	79,522.62	14,493.00	103,610.00	119,377.67	29,400.00
Iqiyi	1,410.98	29,211.41		78,971.72	129,948.00
CCTV	19,349.55	26,806.33	50,423.16	23,632.02	36,386.21
China Central People's Broadcasting and Television Station	347.00	379.00	422.00	590.00	386.00
China Radio and Television International		25.00	75.00	61.00	64.00
Hunan Radio and Television Station	1,085.61	1,639.34	26,655.48	40,010.74	61,620.00
Total	161,755.72	157,703.38	335,185.79	443,556.95	632,597.21

**Table 2:** Classification of CND and broadband fee investment scale.

Unit	2012	2013	2014	2015	2016
Major video sites	0.76	0.67	0.59	0.73	0.71
Major radio and television media	0.02	0.03	0.05	0.02	0.024
Total	0.78	0.70	0.64	0.75	0.74

**Table 3:** HI value of CND and broadband fee investment scale of major video websites and major radio and television media.

Unit	2012	2013	2014	2015	2016
Major video sites	0.76	0.67	0.59	0.73	0.71
Major radio and television media	0.02	0.03	0.05	0.02	0.024
Total	0.78	0.70	0.64	0.75	0.74

**Table 4:** Analysis of HI value of broadband fee investment scale.

Unit	HI value of CND and broadband fee investment scale				
	In 2012	In 2013	In 2014	In 2015	In 2016
Low fusion (1.0–0.84)					
Medium and low fusion (0.84–0.68)	0.78	0.70		0.75	0.74
Moderate fusion (0.68–0.52)			0.64		
Medium-high fusion (0.52–0.36)					
Highly integrated (0.36–0.2)					

**Table 5:** Advertising revenue of major video websites and major radio and television media.

Unit	Advertising revenue (10,000 yuan)				
	In 2012	In 2013	In 2014	In 2015	In 2016
Unity group	142,632.96	167,272.51	280,791.54	295,631.25	335,540.00
Tencent video	4,945.65	11,696.00	235,666.68	400,000.00	599,700.00
Sohu video	55,660.64	13,074.00	110,980.65	103,391.44	100,232.00
Iqiyi	44,598.74	75,278.09	179,755.38	172,111.28	514,785.00
CCTV	25,868.48	24,916.90	34,615.43	28,705.33	38,277.27
China Central People's Broadcasting and Television Station					1,085.57
China Radio and Television International	113.00	664.00	847.00	434.00	696.84
Hunan Radio and Television Station	4,925.45	3,667.18	7,618.66	53,472.86	84,978.00
Total	278,744.92	296,568.68	850,338.34	1,053,746.16	1,675,294.68

**Table 6:** Classification of advertising revenue.

Unit	Advertising revenue (10,000 yuan)				
	In 2012	In 2013	In 2014	In 2015	In 2016
Major video sites	247,837.99	267,320.60	807,194.25	971,133.97	1,550,257.00
Major radio and television media	30,906.93	29,248.08	43,144.09	82,612.19	125,037.68
Total	278,744.92	296,568.68	850,338.34	1,053,746.16	1,675,294.68

**Table 7:** HI value of advertising revenue.

Unit	HI value of advertising revenue				
	In 2012	In 2013	In 2014	In 2015	In 2016
Major video sites	0.79	0.81	0.90	0.85	0.86
Major radio and television media	0.01	0.01	0.003	0.01	0.006
Total	0.80	0.82	0.903	0.86	0.866

**Table 8:** Analysis of HI value of advertising revenue.

Unit	HI value of advertising revenue				
	In 2012	In 2013	In 2014	In 2015	In 2016
Low fusion (1.0–0.84)			0.90	0.86	0.86
Medium and low fusion (0.84–0.68)	0.80	0.82			
Moderate fusion (0.68–0.52)					
Medium-high fusion (0.52–0.36)					
Highly integrated (0.36–0.2)					

**Table 9:** PC page playback.

Unit	PC page playback times (100 million times)				
	In 2012	In 2013	In 2014	In 2015	In 2016
Unity group	1,501.91	1,654.31	1,745.10	1,539.62	3,542.31
Tencent video	783.40	704.68	549.44	400.29	356.08
Sohu video	152.26	201.86	214.39	151.46	622.02
Iqiyi	227.67	295.68	384.00	434.72	251.71
CCTV	300.00	390.00	500.00	450.00	1,519.00
China Central People's Broadcasting and Television Station	32.62	48.44	58.14	41.9	547.33
China Radio and Television International	0.52	0.69	1.30	1.00	0.25
Hunan Radio and Television Station	4.82	5.36	5.20	5.31	5.87
Total	0.63	7.60	32.63	54.95	200.05

**Table 10:** PC client playback.

Unit	PC client playback times (100 million times)				
	In 2012	In 2013	In 2014	In 2015	In 2016
Unity group	1,228.51	1,160.80	1,431.91	1,490.53	1,383.21
Tencent video			77.55	119.60	245.54
Sohu video	269.15	226.37	214.65	166.97	199.54
Iqiyi	341.51	443.52	576.00	652.08	13.46
CCTV	610.00	480.00	550.00	540.00	870.00
China Central People's Broadcasting and Television Station	7.85	10.91	13.72	11.89	14.53
China Radio and Television International					
Hunan Radio and Television Station					
Total					40.15

**Table 11:** Mobile page playback.

Unit	Number of plays on the mobile page (100 million times)				
	In 2012	In 2013	In 2014	In 2015	In 2016
Total	175.86	313.56	1,184.98	2,483.81	3,494.55
Unity group		53.82	114.60	226.50	241.56
Tencent video		1.88	472.36	1,650.64	2,657.01
Sohu video	170.76	221.76	288.00	326.04	137.72
Iqiyi	5.10	36.10	300.00	266.00	340.00
CCTV					35.60
China Central People's Broadcasting and Television Station					
China Radio and Television International			0.43	0.51	2.35
Hunan Radio and Television Station			9.60	14.12	80.30

**Table 12:** Mobile client playback.

Unit	Mobile client playback times (100 million times)				
	In 2012	In 2013	In 2014	In 2015	In 2016
Total	637.34	1,635.54	4,004.29	4,865.63	9,753.45
Unity group	88.91	552.22	1,101.25	1,180.93	1,524.45
Tencent video		112.54	710.38	1,289.79	2,614.28
Sohu video	398.43	517.44	672.00	760.75	227.63
Iqiyi	150.00	450.00	1,500.00	1,500.00	4,871.00
CCTV		3.34	11.06	8.95	33.05
China Central People's Broadcasting and Television Station					1.24
China Radio and Television International					
Hunan Radio and Television Station			9.60	125.21	481.80

**Table 13:** Classification of PC page playback.

Unit	PC page playback times (100 million times)				
	In 2012	In 2013	In 2014	In 2015	In 2016
Total	1,501.91	1,654.31	1,745.10	1,539.62	3,542.31
Major video sites	1,463.32	1,592.22	1,647.82	1,436.47	2,788.81
Major radio and television media	38.58	62.09	97.27	103.16	753.50

**Table 14:** Classification of PC client playback.

Unit	PC client playback times (100 million times)				
	In 2012	In 2013	In 2014	In 2015	In 2016
Total	1,228.51	1,160.80	1,431.91	1,490.53	1,383.21
Major video sites	1,220.66	1,149.89	1,418.19	1,478.64	1,328.53
Major radio and television media	7.85	10.91	13.72	11.89	54.68

**Table 15:** Classification of mobile page playback.

Unit	Number of plays on the mobile page (100 million times)				
	In 2012	In 2013	In 2014	In 2015	In 2016
Total	175.86	313.56	1,184.98	2,483.81	3,494.55
Major video sites	175.86	313.56	1,174.95	2,469.18	3,376.30
Major radio and television media			10.03	14.63	118.26

**Table 16:** Mobile client playback classification.

Unit	Mobile client playback times (100 million times)				
	In 2012	In 2013	In 2014	In 2015	In 2016
Total	637.34	1,635.54	4,004.29	4,865.63	9,753.45
Major video sites	637.34	1,632.21	3,983.63	4,731.47	9,237.36
Major radio and television media	-	3.34	20.66	134.16	516.09

**Table 17:** PC page side playback HI values.

Unit	HI value of PC page playback times				
	In 2012	In 2013	In 2014	In 2015	In 2016
Total	0.95	0.93	0.89	0.87	0.67
Major video sites	0.95	0.93	0.89	0.87	0.62
Major radio and television media	0.001	0.001	0.003	0.004	0.05

**Table 18:** PC client play HI values.

Unit	HI value of PC client playback times				
	In 2012	In 2013	In 2014	In 2015	In 2016
Total	0.99	0.98	0.98	0.98	0.92
Major video sites	0.99	0.98	0.98	0.98	0.92
Major radio and television media	0.00004	0.0001	0.0001	0.0001	0.0016

**Table 19:** Mobile page play HI values.

Unit	HI value of playing times on mobile page side				
	In 2012	In 2013	In 2014	In 2015	In 2016
Total	1.00	1.00	0.98	0.99	0.93
Major video sites	1.00	1.00	0.98	0.99	0.93
Major radio and television media			0.00007	0.00003	0.0011

**Table 20:** Mobile client play HI value.

Unit	HI value of playing times on mobile page side				
	In 2012	In 2013	In 2014	In 2015	In 2016
Total	1.00	1.00	0.99	0.95	0.90
Major video sites	1.00	1.00	0.99	0.95	0.90
Major radio and television media		0.000004	0.000027	0.00076	0.0028

**Table 21:** Calculation results of convergence degree between radio and television and new media.

Project	In 2012	In 2013	In 2014	In 2015	In 2016
Degree of technology integration	0.78	0.70	0.64	0.75	0.74
Market integration	0.80	0.82	0.90	0.86	0.86
Degree of business integration	0.98	0.98	0.96	0.95	0.86

PC page side	0.95	0.93	0.89	0.87	0.67
PC client	0.99	0.98	0.98	0.98	0.92
Move the page side	1.00	1.00	0.98	0.99	0.93
Mobile client	1.00	1.00	0.99	0.95	0.90

**Table 22:** Proportion of CND and broadband fee investment in advertising revenue.

Unit	Specific gravity (%)				
	In 2012 (%)	In 2013 (%)	In 2014 (%)	In 2015 (%)	In 2016 (%)
Major video sites	57	48	32	39	34
Major radio and television media	67	99	180	78	246

**Table 23:** Total play times of play platform.

Unit	Total number of plays (100 million times)				
	In 2012	In 2013	In 2014	In 2015	In 2016
Major video sites	3,497.18	4,687.88	8,224.60	10,115.76	16,731.01
Major radio and television media	46.43	76.34	141.67	263.83	1,442.52

## Data Availability

The data used to support the findings of this study are available from the corresponding author upon request.
